# Promotion of Prescription Drugs to Consumers and Providers, 2001–2010

**DOI:** 10.1371/journal.pone.0055504

**Published:** 2013-03-04

**Authors:** Rachel Kornfield, Julie Donohue, Ernst R. Berndt, G. Caleb Alexander

**Affiliations:** 1 Section of General Internal Medicine, Department of Medicine, University of Chicago, Chicago, Illinois, United States of America; 2 Department of Health Policy and Management, University of Pittsburgh, Pittsburgh, Pennsylvania, United States of America; 3 Department of Psychiatry, University of Pittsburgh, Pittsburgh, Pennsylvania, United States of America; 4 Alfred P. Sloan School of Management, Massachusetts Institute of Technology, Cambridge, Massachusetts, United States of America; 5 National Bureau of Economic Research, Cambridge, Massachusetts, United States of America; 6 Department of Epidemiology, Johns Hopkins Bloomberg School of Public Health, Baltimore, Maryland, United States of America; 7 Department of Medicine, Johns Hopkins Medicine, Baltimore, Maryland, United States of America; 8 Department of Pharmacy Practice, University of Illinois at Chicago School of Pharmacy, Chicago, Illinois, United States of America; University of Milan, Italy

## Abstract

**Background:**

Pharmaceutical firms heavily promote their products and may have changed marketing strategies in response to reductions in new product approvals, restrictions on some forms of promotion, and the expanding role of biologic therapies.

**Methods:**

We used descriptive analyses of annual cross-sectional data from 2001 through 2010 to examine direct-to-consumer advertising (DTCA) (Kantar Media) and provider-targeted promotion (IMS Health and SDI), including: (1) inflation-adjusted total promotion spending ($ and percent of sales); (2) distribution by channel (consumer v. provider); and (3) provider specialty both for the industry as a whole and for top-selling biologic and small molecule therapies.

**Results:**

Total promotion peaked in 2004 at US$36.1 billion (13.4% of sales). By 2010 it had declined to $27.7B (9.0% of sales). Between 2006 and 2010, similar declines were seen for promotion to providers and DTCA (both by 25%). DTCA’s share of total promotion increased from 12% in 2002 to 18% in 2006, but then declined to 16% and remains highly concentrated. Number of products promoted to providers peaked in 2004 at over 3000, and then declined 20% by 2010. In contrast to top-selling small molecule therapies having an average of $370 million (8.8% of sales) spent on promotion, top biologics were promoted less, with only $33 million (1.4% of sales) spent per product. Little change occurred in the composition of promotion between primary care physicians and specialists from 2001–2010.

**Conclusions:**

These findings suggest that pharmaceutical companies have reduced promotion following changes in the pharmaceutical pipeline and patent expiry for several blockbuster drugs. Promotional strategies for biologic drugs differ substantially from small molecule therapies.

## Introduction

In the United States, pharmaceuticals are heavily promoted to providers and patients. The pharmaceutical industry spent nearly $30 billion dollars in 2005 on marketing and promotion, of which 84% went toward physician detailing and free samples, with less devoted to professional advertising and direct-to-consumer advertising (DTCA) [1], [2]. Spending varied considerably by product, although both detailing and DTCA tended to favor drugs with broader clinical indications for use [3]. Pharmaceutical promotion can influence demand for prescription drugs [4], increase physician visits for conditions treated by heavily advertised drugs [5] and affect physician prescribing [6].

Little is known about how pharmaceutical companies have altered promotional spending in response to major health care changes. First, during the past decade there has been a slowdown in new drug introductions. During the second half of the 1990s, the FDA approved a large number of small molecule therapies for common conditions, including many drugs that were the first of their kind. These “blockbuster” drugs were heavily marketed, resulting in a 162% increase in total promotional spending between 1996 and 2005 [1]. In recent years, however, blockbuster drugs have faced increasing competition from generics, as well as branded rivals, with the generic share of total prescriptions increasing markedly from 63% in 2006 to nearly 80% in 2010 [7]. Fewer new drugs have been approved annually in recent years [8], and a greater proportion of those introduced have been for orphan conditions [9]. Second, drugs manufactured using biologic processes, or “biologics”, represent an increasing proportion of newly approved products and drugs sales [10], [11]. Biologics comprised over 40% of products in late stage research and development in 2009, suggesting that they may account for an increasing proportion of new products launched in the near future [10]. Since these products are often used by a smaller number of patients, administered parenterally by providers, and sold at much higher prices, the promotional strategies may differ substantially compared to small molecule therapies. Finally, in response to mounting empirical evidence as well as legal challenges, media scrutiny [12], and the recommendations of professional societies [13], numerous medical centers have limited pharmaceutical sales representatives access to physicians [14]–[16]. Furthermore, certain states now require disclosure of gifts from pharmaceutical companies to providers [17]. While there is some evidence of decreases in industry interaction with office-based physicians [18], [19], it is unclear how industry practices have changed in response to these provisions.

We examined trends in promotion to consumers and providers over the last decade. We hypothesized decreases in absolute spending on promotion to providers and DTCA, with an increasing share of detailing devoted to specialists given the expanding role of biologics. In addition to trends for the pharmaceutical industry overall, we compared the promotional strategies of top-selling small molecule and biologic therapies. Finally, to determine whether trends in promotion were correlated with changes in the pharmaceutical pipeline, we examined the number of products and spending per product promoted.

## Methods

### Data

We used the IMS Health Integrated Promotional Services™ to obtain data on detailing, free samples dispensed to providers, and journal advertisements. We obtained data from SDI on spending for electronic promotion (e.g., Internet) targeting providers and for meetings and conferences. IMS Health detailing estimates are derived from a nationally representative audit of office- and hospital-based providers as well as pharmacy directors. Office-based detailing includes spending on service visits associated with sample distribution. Estimates of units of free samples dispensed to physicians are derived from an audit of office-based physician practices, while their retail value is calculated based on suggested retail prices. Journal advertising data is collected through a census of all medical journals. Using directory information from the American Medical Association, IMS also reports detailing expenditures by physician specialty. SDI spending is based on a monthly audit of approximately 4,000 office-based providers representing 19 specialties. Data are collected and projected by region and specialty to represent a universe of approximately 380,000 practicing providers. Finally, Kantar Media provided industry-wide and product-specific DTCA expenditures accounting for television, magazine, radio, outdoor, newspaper, and Internet promotion. These estimates are drawn from a sample of national media such as network TV and national newspapers as well as local media sampled at the Designated Media Area level.

We used IMS Health sales figures [7], supplemented for certain therapies with data from the IMS Health National Sales Perspectives™, in order to calculate promotion and marketing as a percentage of total sales. Estimates of the annual sales were calculated based on unit sales from both retail and non-retail channels and ex-manufacturer invoices (amount paid to wholesalers or manufacturers net of prompt payment discounts). We obtained data on the number of products on the market and, of these, the number promoted each year using IMS Health National Sales Perspectives™ and Integrated Promotional Services™. We used a data set of drug launches [10], supplemented for 2009 and 2010 with the number of new molecular entities approved by the Food and Drug Administration [20], to determine the number of new molecular entities per year.

Biologic therapies were defined as those manufactured using biologic processes [10], while the remainder of products were categorized as small molecules.

### Analyses

We used descriptive statistics to characterize six aspects of promotion to providers: the retail value of free samples, office-based detailing, hospital-based detailing, journal advertising, epromotion and conferences and meetings. We quantified the absolute and relative magnitude of annual total promotional efforts towards providers. We also assessed the concentration of promotion for top-selling small molecules and biologic therapies.

We obtained a list of the top-selling U.S. and European biologics in 2010 [21]. We then identified additional biologics with high sales expenditures [22] and used the IMS Health National Sales Perspectives™ to rank these therapies. Sales and promotional expenditures were aggregated across all formulations of a brand, and for the few molecules available both as monotherapies and fixed-dose combinations, we excluded sales and promotional spending associated with combination therapies. Except where otherwise noted, data on sales and promotional spending were adjusted to 2010 dollars using the Consumer Price Index – All Urban [23].

## Results

### Trends in Overall and Provider Promotion

Table 1 characterizes aggregate trends in marketing and promotion. Total inflation-adjusted promotional spending peaked in 2004 both in terms of absolute spending ($36.1 billion) and spending relative to sales (13.4%). Afterward, spending declined each year to $27.7B (9.0% of sales) by 2010. Nearly all forms of promotion saw declines beginning in 2005. The retail value of free samples declined 23%, or 11% when not adjusted for inflation, from $18.1 B in 2004 to $13.9B in 2010. The expenditure shares across the three major promotional categories were remarkably stable. Despite a more than two-fold relative increase in electronic promotion, this category accounted for less than 2% of provider promotion in 2010.

**Table 1:** Pharmaceutical promotion to consumers and providers 2001–2010.

	2001	2002	2003	2004	2005	2006	2007	2008	2009	2010
Direct-to-consumer advertising (millions of 2010 dollars)										
Television	2,184	2,061	2,367	3,213	3,150	3,270	3,194	2,951	2,919	2,375
Print	1,242	1,242	1,606	1,651	1,823	2,291	2,132	1,617	1,587	1,747
Internet	27	42	72	214	181	230	105	141	312	202
Radio	46	51	73	67	68	87	48	24	43	44
Outdoor	2	6	6	6	8	13	4	3	6	3
Total	3,500	3,402	4,124	5,151	5,231	5,891	5,483	4,738	4,868	4,371
As percentage of sales	1.7	1.4	1.6	1.9	1.9	2.0	1.9	1.6	1.6	1.4
Promotion to providers (millions of 2010 dollars)										
Office-based promotion	5,897	6,450	7,442	7,621	6,892	6,780	6,147	6,043	5,906	5,306
Hospital-based promotion	864	1,071	1,005	1,059	881	718	620	490	491	479
Journal advertising	523	578	582	628	531	570	494	392	320	326
Free samples (retail value)	12,884	14,455	16,057	18,056	16,318	14,970	15,614	14,193	14,416	13,850
Epromotion (SDI)	–	–	251	255	314	356	415	497	532	525
Conferences and meetings (SDI)	2,605	2,644	2,890	3,295	3,027	2,851	2,910	2,993	2,952	2,840
Total	22,773	25,197	28,229	30,915	27,963	26,242	26,201	24,609	24,616	23,326
As percentage of sales	10.8	10.7	10.9	11.4	10.1	9.0	8.9	8.5	8.1	7.6
All DTCA and promotion to providers ($2010 millions)	26,274	28,599	32,352	36,065	33,194	32,133	31,685	29,347	29,484	27,697
All sales ($2010 billions)	212	236	260	270	276	292	296	290	305	307
As percentage of sales	12.4	12.1	12.5	13.4	12.0	11.0	10.7	10.1	9.7	9.0
Number of new molecular entities launched	31	28	30	21	20	27	21	19	26	21
Number of products marketed and promoted	2,920	3,087	3,056	3,105	3,094	2,680	2,730	2,660	2,576	2,474
Average promotion per product ($millions)	9.0	9.3	10.6	11.6	10.7	12.0	11.6	11.0	11.4	11.2

All financial data were adjusted to 2010 dollars, utilizing the Consumer Price Index – All Urban.

Sources: Direct-to-consumer advertising data provided by Kantar Media; promotion to professionals data derived from the IMS Health Integrated Promotional Services™, 2002–2010 with the exception of data regarding epromotion and conferences and meetings which was derived from the SDI Physician Meeting and Event Audit and SDI ePromotion Audit; provider promotion for 2001 derived from reference #1; sales data derived from IMS Health Use of Medicines 2010 Report; newly launched molecular entities derived from reference #10; number of products marketed and promoted derived from IMS Health Integrated Promotional Services™ and includes products with any spending targeting providers.

### Trends in Direct-to-consumer Advertising (DTCA)

DTCA peaked at $5.9B in 2006 followed by a 25% decline to $4.4B by 2010. As a percentage of total promotional spending, DTCA increased from 12% in 2002 to 18% in 2006, but declined modestly to 16% by 2010. During this period, television accounted for a decreasing proportion of all DTCA, declining from 62% in 2001 to 54% by 2010. Print DTCA increased 84% 2001–2006, but then declined 24% by 2010. In 2010, internet promotion accounted for less than 5% of overall consumer promotion.

### Drug Launches and Overall Number of Products Promoted

The number of new molecular entities launched ranged from 19 to 31 across the study period, with the greatest numbers of new molecular entities introduced between 2001 and 2003 (Table 1). Declines in the number of products promoted paralleled declines in promotional spending. The average promotional spending per product actually increased from $9.0M (2001) to $12.0M (2006), then declined modestly to $11.2M (2010).

### Promotion of Top-selling Agents

Among the 25 top-selling products of 2010 listed in Table 2, 16 were small molecule therapies and the remaining nine were biologics.

**Table 2:** U.S. sales revenue and promotional spending for leading selling prescription medicines according to dollar sales in 2010.

Rank	Therapy	Type of therapy	U.S. Sales (billions)	Promotion (millions)							Percentage of sales
				DTCA	Office	Hospital	Samples	Journals	All Provider	Total	
1	Lipitor	Small molecule	7.2	272.0	97.3	7.6	359.7	4.3	468.8	740.8	10.3%
2	Nexium	Small molecule	6.4	16.7	32.5	2.3	208.5	0.7	244.0	260.7	4.1%
3	Plavix	Small molecule	6.1	127.3	60.1	9.1	93.3	0.2	162.7	290.0	4.8%
4	Seroquel	Small molecule	5.2	80.6	51.2	11.8	91.0	0.0	153.9	234.5	4.5%
5	Advair Diskus	Small molecule	4.7	200.5	47.5	1.8	343.4	0.0	392.7	593.2	12.6%
6	Abilify	Small molecule	4.6	155.7	49.7	6.1	412.7	0.0	468.5	624.2	13.6%
7	Singulair	Small molecule	4.1	70.3	69.5	3.6	309.5	0.04	382.6	452.9	11.0%
8	Crestor	Small molecule	3.8	95.3	101.5	7.0	389.7	1.0	499.2	594.5	15.6%
9	Actos	Small molecule	3.5	40.7	48.9	1.5	202.2	0.0	252.6	293.3	8.4%
10	Epogen	Biologic	3.3	0	0.4	0.1	0.0	0.0	0.4	0.4	0.01%
11	Remicade	Biologic	3.3	0	4.7	0.7	0.3	0.6	6.3	6.3	0.2%
12	Enbrel	Biologic	3.3	71.5	9.9	0.9	8.1	1.2	20.1	91.6	2.8%
13	Zyprexa	Small molecule	3.3	1.2	16.0	5.8	174.1	0.0	195.9	197.1	6.0%
14	Cymbalta	Small molecule	3.2	206.0	93.6	7.2	309.6	4.0	414.4	620.4	19.4%
15	Avastin	Biologic	3.1	0.0007	2.8	1.6	0.0	2.2	6.6	6.6	0.2%
16	Oxycontin	Small molecule	3.1	0.1	9.9	0.9	0.0	2.6	13.4	13.5	0.4%
17	Lantus	Biologic	3.0	46.5	37.2	4.7	58.3	8.3	108.5	154.9	5.1%
18	Neulasta	Biologic	3.0	0.3	1.4	0.2	0.0	0.7	2.3	2.6	0.1%
19	Humira	Biologic	2.9	34.1	12.9	3.8	25.4	0.1	42.2	76.3	2.6%
20	Lexapro	Small molecule	2.8	2.1	108.2	6.7	270.9	13.1	398.8	400.9	14.3%
21	Rituxan	Biologic	2.8	0.05	4.3	0.2	0.0	2.3	6.8	6.9	0.2%
22	Aricept	Small molecule	2.5	34.3	25.5	2.6	154.1	2.2	184.5	218.8	8.8%
23	Lovenox	Small molecule	2.3	0.1	7.3	8.5	3.2	0.0	19.0	19.1	0.8%
24	Atripla	Small molecule	2.2	0.8	2.1	1.0	0.2	0.4	3.7	4.5	0.2%
25	Copaxone	Biologic	2.2	0	4.0	0.7	2.3	0.2	7.2	7.2	0.3%
TOTAL	–	–	91	1,456	20%	2%	77%	1%	4,455	5,911	6.4%

Sources: Direct-to-consumer advertising data provided by Kantar Media; promotion to professionals data derived from the IMS Health Integrated Promotional Services™, 2010™ and excludes epromotion and expenditures for conferences and meetings depicted in Table 1; sales data derived from IMS Health Use of Medicines 2010.

Levels and intensities of provider and consumer-directed promotion were generally lower for biologics than small molecule therapies. The top 15 small molecule therapies had an average total promotional spending of $370 million in 2010 (8.8% of sales) compared to only $33 million for the top 15 biologics (1.4% of sales).

### Products Most Heavily Promoted to Consumers

Table 3 displays the 25 drugs most heavily promoted to consumers via DTCA. The drug most heavily promoted to consumers in 2010 was Lipitor with $272M devoted to DTCA alone followed by Cialis ($216M) and Cymbalta ($206M). DTCA was concentrated in a small number of products. Only two of the top 25 consumer-promoted products, etanercept (Enbrel) and golimumab (Simponi), were biologic therapies, whereas biologics accounted for 9 of the 25 top-selling products.

**Table 3:** Therapies most heavily promoted through direct-to-consumer advertising, 2010.

Ranking	Trade name	Type of drug	Spending in direct-to-consumer advertising (millions)
1	Lipitor	Statin	272
2	Cialis	Phosphodiesterase type 5 inhibitor	216
3	Cymbalta	Serotonin-norepinephrine reuptake inhibitor	206
4	Advair	Inhaled corticosteroid and long-acting beta-agonist	200
5	Abilify	Atypical antipsychotic	156
6	Symbicort	Inhaled corticosteroid and long-acting beta-agonist	152
7	Pristiq	Serotonin-norepinephrine reuptake inhibitor	127
8	Plavix	Oral thienopyridine antiplatlet	127
9	Lyrica	Anticonvulsant	112
10	Chantix	Nicotinic receptor partial agonist	110
11	Toviaz	Muscarinic antagonist	109
12	Viagra	PDE5 inhibitor	100
13	Crestor	Statin	95
14	Boniva	Oral bisphosphonate	85
15	Lovaza	Omega-3 fatty acid	81
16	Seroquel	Atypical antipsychotic	81
17	Enbrel*	Tumor necrosis factor inhibitor	72
18	Simponi*	Tumor necrosis factor inhibitor	71
19	Spiriva Handihaler	Anticholinergic bronchodilator	71
20	Singulair	Leukotriene receptor antagonists	70
21	Januvia	Dipeptidyle peptidase-4 (DPP-4) inhibitor	65
22	Restasis	Cyclosporin topical emulsion	58
23	Vyvanse	Psychostimulant	58
24	Trilipix	Fibrate	56
25	Lunesta	Non-benzodiazepine hypnotic	54
All 25 combined			2,805
Total percentage of industry DTCA spending			64

Source: Data provided by Kantar Media.

* Biologic therapy.

### Promotion of Biologics

Table 4 reports top US-selling biologics along with product-specific expenditures and promotional spending toward consumers and providers. In 2010, epoetin alfa (Epogen), infliximab (Remicade) and etanercept (Enbrel) led in biologic sales, each with $3.3B. Among top-selling biologic therapies, 2010 promotion was greatest for exenatide (Byetta) with 20% of its $571M in US sales dedicated to promotion, followed by insulin detemir (Levemir) with 12% and insulin glargine (Lantus) with 5% of its $3.0B in U.S. sales dedicated to promotion. Promotion for 17 of the other top-selling 25 biologics was less than 1% of sales.

**Table 4:** U.S. sales revenue and promotional spending for leading selling biologics according to dollar sales in 2010.*

Rank	Therapy	U.S. Sales (millions)	Promotion			Percentage of sales	Type of provider promotion (thousands)			
			DTCA (thousands)	Provider (thousands)	Total(thousands)		Office	Hospital	Samples	Journals
1	Epogen	3,325	0	447	447	0.01%	394	53	0	0
2	Remicade	3,303	0	6,270	6,270	0.2%	4,682	679	277	632
3	Enbrel	3,291	71,507	20,129	91,636	2.8%	9,864	931	8,143	1,192
4	Avastin	3,091	1	6,643	6,644	0.2%	2,837	1,570	0	2,237
5	Lantus	3,045	46,461	108,474	154,935	5.1%	37,178	4,696	58,284	8,316
6	Neulasta	3,011	252	2,291	2,543	0.1%	1,379	217	0	695
7	Humira	2,929	34,108	42,206	76,314	2.6%	12,894	3,778	25,390	144
8	Rituxan	2,762	45	6,780	6,825	0.2%	4,314	202	0	2,264
9	Copaxone	2,253	0	7,177	7,177	0.3%	3,983	723	2,256	216
10	NovoLog	2,097	4,496	53,130	57,626	2.7%	11,261	890	39,566	1,413
11	Humalog	1,608	13,665	57,805	71,470	4.4%	13,075	1,037	35,671	8,022
12	Herceptin	1,537	0	2,563	2,563	0.2%	1,544	264	0	754
13	Procrit/Eprex	1,466	13	2,277	2,290	0.2%	1,295	867	0	115
14	Lucentis	1,435	2,053	666	2,719	0.2%	274	53	0	339
15	Avonex	1,424	334	4,231	4,565	0.3%	2,965	487	258	521
16	Aranesp	1,305	0	3,470	3,470	0.3%	1,971	1,499	0	0
17	Neupogem	961	0	83	83	0.01%	74	9	0	0
18	Rebif	941	92	4,439	4,531	0.5%	3,952	41	0	446
19	Prevnar-7	829	16,277	6,851	23,128	2.8%	4,611	395	0	1,845
20	Betaseron	826	4	3,148	3,152	0.4%	2,857	20	0	271
21	Synagis	735	0	2,910	2,910	0.4%	2,181	728	0	0
22	Erbitux	709	0	3,640	3,640	0.5%	2,318	191	0	1,131
23	Levemir	673	144	82,889	83,033	12.3%	27,125	2,782	48,242	4,740
24	Byetta	571	42	113,461	113,503	19.9%	23,121	1,598	85,194	3,549
25	Pegasys	512	0	3,447	3,447	0.7%	3,016	431	0	0
TOTAL	–	44,639	189,494	545,427	734,921	1.6%	33%	4%	56%	7%

Sources: Direct-to-consumer advertising data provided by Kantar Media; promotion to professionals data derived from the IMS Health Integrated Promotional Services™, 2010 and excludes epromotion and expenditures for conferences and meetings depicted in Table 1; sales data derived from IMS National Sales Perspectives™.

Spending on promotion to providers varied widely across the biologics examined, ranging from only $83,000 (filgrastim [Neupogen]) to more than $100 million (insulin glargine [Lantus] and exenatide [Byetta]). For the majority of therapies, office-based detailing accounted for the largest expenditures; however, among the minority of biologics that had any spending on free samples (e.g., Byetta, Lantus, Levemir), this was generally the dominant form of promotion. DTCA for biologics was limited to approximately two-thirds of the 25 therapies examined.

### Promotion to Primary Care Physicians and Specialists

Table 5 summarizes trends in detailing and contacts directed at primary care providers and specialists (excluding free samples). The proportion of office-based detailing directed at primary care providers declined modestly from 69% of contacts in 2002 to 63% in 2010. However, smaller decreases were evident in the share of office-based detailing spending targeting primary care physicians.

**Table 5:** Detailing spending and number contacts with primary care providers and specialists 2001–2010.

	2001	2002	2003	2004	2005	2006	2007	2008	2009	2010
Spending on Office-Based Detailing										
Primary Care, %	–	62.0	–	62.3	61.9	61.0	60.9	60.5	60.6	60.3
Specialty, %	–	38.0	–	37.7	38.1	39.0	39.1	39.5	39.4	39.7
Total (millions $2010)	5,897	6,450	7,442	7,621	6,892	6,780	6,147	6,043	5,906	5,306
Office-based Contacts										
Primary Care, %	69.3	68.6	–	68.5	67.7	63.2	63.1	62.4	62.8	62.6
Specialty, %	30.7	31.4	–	31.5	32.3	36.7	36.9	37.5	37.2	37.3
Total (millions)	50.8	53.6	67.7	69.0	60.1	58.8	54.0	51.9	48.9	44.6

All data were adjusted to 2010 dollars, utilizing the Consumer Price Index. Primary care providers include those trained in family practice, general practice, internal medicine, osteopathic medicine or pediatrics. Specialty providers were defined as all other provider types, including those trained in subspecialties of internal medicine such as cardiology or gastroenterology.

“–” indicates years when data was not available.

Source: IMS Health Integrated Promotional Services™, 2001–2010.

## Discussion

After steady increases in pharmaceutical marketing and promotion to consumers and providers during the first half of the last decade, since 2004 pharmaceutical firms have decreased both the absolute value of spending as well as the share of sales devoted to promotion. These declines in promotional spending do not seem to primarily reflect waning consumer purchasing power, since promotion has been declining in the context of rising sales [7]. Spending on meetings and electronic promotion has increased, yet these channels still account for only a small fraction of provider promotion. Despite its growth in the first half of the decade, DTCA also represents a minority of promotion and is driven by television advertising. Top-selling biologic therapies had far lower promotional spending per product than did the top small molecule therapies, with substantially less spent on free samples.

Declines in promotion as a percentage of sales since 2005 may result in part from the “graying” of the market [1]. Whereas sales for new drugs accounted for 34% of total sales in 1999 they comprised only 19% of total sales in 2007 [8]. Reductions in new molecular entity approvals are apparent when considering the 1990s. On average, 22 new molecular entities were introduced annually in the 1980s, 31 in the 1990s, and 24 in the 2000s [24].

Declining promotion may also reflect the increasing biologics share of the market [10]. Biologics often have unique routes of delivery and storage and can be very costly compared to small molecules, with costs for one cancer drug, Avastin, exceeding $100,000 per year [25]. Given that use of new biologics is concentrated among a smaller number of patients with relatively rare conditions treated primarily by specialists, we would expect promotion to providers and consumers to also be highly targeted.

Despite anecdotal reports [26], [27] and calls from stakeholders [27]–[29], we did not find evidence of substantial changes in the proportion of provider-targeted promotion accounted for by office-based detailing. In addition, we saw no substantial shifts in the proportion of expenditures targeting primary care providers.

DTCA remains highly concentrated among a small number of products and continues to account for a minority of promotional spending [30]. Declines in DTCA may accelerate as biologics make up a greater share of new therapies. Although relative increases in DTCA through media such as the Internet and social networking have occurred, these expenditures remain a small fraction of overall consumer-targeted promotion.

Our study has several limitations. First, our analyses were not designed to examine promotional content nor the causal effect of promotional expenditures [31]–[33]. Second, some biologics have unique distribution channels and thus our data capture may be incomplete. The difficulty in measuring the extended units for infused and injected therapies also prohibits us from estimating the ratio of promotion to units of utilization. Third, while there are a variety of methods of estimating promotion costs [34], we have used a conventional commercial definition and have considered only expenditures that are clearly directed at marketing rather than attempting to approximate unmonitored promotion and the R&D proportion that is promotional. Our estimates are similar to those of Donohue et al [1] although here we include estimates of expenditures for conferences and meetings as well as Epromotion to providers. As with prior investigations [1], our estimations of promotion devoted to free samples are based on their approximate retail value and thus may overstate manufacturers’ costs. Finally, to the extent medical care prices have increased more rapidly than non-medical care prices, our use of the Consumer Price Index – All Urban may underestimate the magnitude of the reduction in inflation-adjusted drug spending since 2006.

Manufacturers of branded pharmaceuticals continue to expend considerable sums on promotion to consumers and providers. However, in the context of marketplace changes, firms are decreasing spending but changing little about how expenditures are allocated across types of promotion. An increasing role for biologics to the market may cause more substantial shifts in future promotional patterns.
